# A Predictive Model for the Risk of Cognitive Impairment in Patients with Gallstones

This article has been retracted.

**DOI:** 10.1155/2021/3792407

**Published:** 2021-07-17

**Authors:** Zhaofang Liu, Chuanyan Li

**Affiliations:** Department of General Surgery, The First Affiliated Hospital of USTC, China

## Abstract

**Objectives:**

Gallstones can cause malnutrition in patients and further lead to cognitive impairment. This study is aimed at constructing a validated clinical prediction model for evaluating the risk of developing cognitive impairment from gallstones.

**Methods:**

The study was a single-centre crosssectional study. Four models or methods (SVM-RFE, random forest model, Lasso model, and logistics analysis) were analyzed and compared regarding their predictive performance. The model with the best classification performance and predictive power was selected. The AUC index, C-index, and calibration curves were applied to the chosen model to further evaluate its classification and prediction performance. Finally, the nomogram was plotted, and the clinical usability, efficacy, and safety of the nomogram were assessed using decision curve analysis (DCA).

**Results:**

This study included a total of 294 patients with gallstones, of which 110 had cognitive impairment. Factors such as gender, age, education, place of birth, history of alcohol consumption, abdominal circumference, sarcopenia, diabetes, anaemia, depression, and Pittsburgh Sleep Quality Index (PSQI) were incorporated into the model for nomogram construction. The calibration curve showed that the nomogram had good classification performance. Furthermore, the C-index of the model was 0.778 (95% CI, 0.674-0.882) in the test group. The DCA curves indicated that the constructed model had strong clinical applicability, efficacy, and safety.

**Conclusions:**

This study constructed a cognitive impairment risk prediction model for patients with gallstones with good classification and predictive power. The constructed predictive model allows us to screen patients with gallstones and at high risk of cognitive impairment. These efforts might also help to further increase patient compliance, assist healthcare professionals to better manage patients with gallstones, and ultimately improve their overall health status and quality of life. Future clinical studies should further evaluate the accuracy and clinical usability of this model.

## 1. Introduction

Although most gallstone carriers are asymptomatic, up to 20% of adults develop gallstones at some point in their lives, and more than 20% of these patients have complications [1, 2]. The known risk factors for gallstones are getting older, pregnancy, lack of physical activity, obesity, and metabolic changes such as overnutrition [1]. Gallstones and cognitive disorders can cause anorexia, leading to weight loss, malnutrition, and other problems [3]. Malnutrition also plays a role in the development of sarcopenia [4]. This finding is in agreement with a meta-analysis study, showing that the prevalence of sarcopenia was between 41% and 46% in older people (aged >60 years), with malnutrition being an independent risk factor [5]. In addition, several studies have revealed that sarcopenia is also a risk factor for cognitive impairment and cognitive impairment [6, 7]. By reducing appetite, cognitive impairment can continue to exacerbate the severity of malnutrition. Thus, cognitive impairment and malnutrition usually operate in a vicious cycle. Treatment of gallstones is still predominantly invasive and relies mainly on surgery [1]. Cognitive impairment is considered to be an important factor that hinders patients from undergoing surgery [8]. Hence, it is important to examine the risk factors associated with cognitive impairment in patients with gallstones. This would help healthcare professionals manage the disease in patients with gallstones, allowing them to make appropriate and timely surgical decisions.

Previous studies have indicated that the prevalence of cognitive impairment in older people (aged ≥65 years) is between 5% and 10%. Various factors are known to be associated with cognitive impairment, including hypertension, diabetes, anaemia, cerebrovascular disease, smoking, alcohol consumption, and lack of exercise [9–12]. A closer look at the literature on risk factors for cognitive impairment, however, reveals a number of gaps and shortcomings. Namely, there is a lack of systematic assessment and, in particular, a lack of knowledge of risk factors for cognitive impairment in patients with gallstones. Thus, a risk prediction tool is needed for assessing risk factors and visualizing the results to solve these problems. Previous studies have suggested that nomogram-based clinical prediction models can be employed to assist clinicians in visually calculating and assessing the incidence of disease for each patient [13, 14]. The development of a clinical risk prediction tool requires the collection of raw data and the extensive screening of clinical characteristics and models. However, a number of scales already exist that can be used for cognitive impairment, such as the Mini-Mental State Examination (MMSE) and Clinical Dementia Rating (CRD) [15, 16]. By using these scales together, a specialist psychiatrist can easily make a diagnosis of cognitive impairment. We, therefore, hypothesized that a valid predictive model could be developed to predict the likelihood of cognitive impairment in people with gallstones based on clinical and epidemiological characteristics and these scoring scales for cognitive impairment.

This study is aimed at building a nomogram prediction model for cognitive impairment in patients with gallstones. The model is expected to lead to more proper psychiatric care for patients. This study also sheds light on the importance of care and social support for elderly cognitive impairment patients with gallstones.

## 2. Materials and Methods

### 2.1. Patients

We selected patients diagnosed with gallstones at the First Affiliated Hospital of USTC from January 2018 to January 2021 for a crosssectional study. Inclusion criteria were age > 60 years, documented preoperative, and absence of any organ failure. Exclusion criteria were patients with malignant diseases such as gallbladder cancer, patients taking relevant psychotropic drugs, and patients with missing clinical features of the relevant study or no outcome indicators recorded. This study was approved by our institutional ethics committee, and informed consent was obtained from the patients.

### 2.2. General Clinical Data of the Patients

The medical case record data included demographic and clinically relevant information on the patients. Demographic information, including sex, age, abdominal circumference, BMI, marital status, educational attainment, smoking history, alcohol history, place of birth, and exercise status, was collected. The data on clinical characteristics include heart rate, hypertension, sarcopenia, diabetes, and anaemia, as well as psychosocial score ratings such as depression status and social impact scores. History and demographic data on hypertension, diabetes mellitus, and anaemia were collected through medical records. Patients were also contacted via telephone if there were missing values. The diagnosis of sarcopenia was based on the Asian Working Group for Sarcopenia (AWGS) 2019 consensus: sarcopenia is diagnosed as a loss of muscle mass and a reduction in muscle strength and somatic function [17].

### 2.3. Diagnosis of Cognitive Impairment and Related Psychiatric Diagnoses

The Mini-Mental State Examination (MMSE) scale was used to screen cognitive impairment. The selection of relevant thresholds was consistent with previous studies in the literature [16]. The Clinical Dementia Rating (CDR) Scale was also used to evaluate the mental status of the patients [15, 18]. The Hamilton Rating Scale for Depression (17-item version, HAMD-17) was employed to measure the severity of depression in patients with gallstones who had not undergone surgical treatment [19]. Patients with a total score of ≥8 on the HAMD-17 were identified as having depression [20].

### 2.4. Other Social Behaviour Assessment Scales

The Pittsburgh Sleep Quality Index (PSQI) was used to evaluate the quality of sleep in patients with gallstones [21]. PSQI scores range from 0 to 21, with higher scores representing poorer sleep quality. It is important to note that the internal consistency of the PSQI measured by Cronbach's alpha is excellent [22]. The Social Impact Scale (SIS) was used to evaluate patients' psychological coping skills in response to social stigma [23]. The European Organisation for Research and Treatment of Cancer's (EORTC) Quality of Life Questionnaire (QLQ-C30) was performed to assess the quality of life of patients with gallstones and tumours, bearing in mind that both groups of patients suffer from chronic diseases. Core 30 (QLQ-C30) was also employed to evaluate the quality of life of patients [24, 25]. It must be stated that a higher score on this scale indicates a poorer quality of life.

### 2.5. Predictive Model and Predictor Screening

Patients were randomly divided into training and validation groups in a ratio of 2 : 1. The training group was used to train the parameters of each model. On the other hand, the validation group was used to validate and compare the performance of each prediction model. A total of four models or methods were applied for predictive model construction, namely, the random forest model, SVM-RFE, Lasso model, and logistics analysis. The model with the strongest predictive power was selected based on its AUC value. The random forest model has several advantages, including its handling of high-dimensional data, the ability to build predictive models, and the ability to estimate the importance of each variable [26]. Support Vector Machine-Recursive Feature Elimination (SVM-RFE) is advantageous for small sample size datasets [27]. The SVM-RFE also has the ability to remove redundant factors and retain only the outcome related variables. The least absolute shrinkage and selection operator (Lasso) regression analysis is often employed to filter variables to prevent overfitting [28]. It uses the default tenfold crossvalidation. Multifactor logistic regression models are created for the screened variables based on the lambda.min value corresponding to the smallest loss. These analyses (both univariate and multifactorial logistic analyses) are often performed in medical research to screen for independent prognostic factors. Factors with *P* < 0.1 on the univariate logistic analysis were included in the multifactor logistic analysis. Similarly, the factors were further filtered by *P* < 0.1 in the subsequent multifactor logistic analyses. The final filtered variables were subjected to multifactor logistics prediction model construction.

### 2.6. Nomogram Validation

AUC values were calculated to evaluate each model's classification performance, and ROC curves were plotted for visualisation. Finally, the model with the highest AUC value was selected for nomogram plotting and further evaluation [13, 14]. Correction curves were plotted for visualising the model prediction accuracy. The C-index was calculated to quantitatively assess the model prediction accuracy. DCA curves were plotted to judge the clinical usability and safety of the model [29].

### 2.7. Statistical Analysis

R software (version 3.5.3) was employed for all statistical analyses. Two-tailed *t*-tests were used for significance testing of continuous variables. Pearson chi-square tests were used for categorical variables. For all statistical tests, a *P* < 0.05 was considered to be statistically significant.

## 3. Results

### 3.1. Patient Demographics and Clinical Characteristics

Figure 1 depicts the flow chart and patient inclusion process. A total of 294 patients with gallstones (192 females and 102 males) were included in the study, of whom 110 had been previously diagnosed with cognitive impairment.  Table 1 reveals the differences between the general and clinical characteristics of patients with or without cognitive impairment. Factors such as age, gender, sarcopenia, education, history of alcohol consumption, the prevalence of diabetes, proportion of anaemia, frequency of exercise, proportion of depression, and PSQI scores were statistically significantly different between the two groups (*P* < 0.05). However, there were no statistical differences in factors such as BMI, heart rate, marital status, place of birth, smoking history, hypertension history, health insurance status, Social Impact Scale score, and total score of QLQ-C30 (*P* > 0.05).

### 3.2. Predictive Model and Predictor Screening

Figures 2 and 3 exhibit the model screening process. The SVM-RFE model has nonlinear discriminatory properties, which allows the comparison of results after modelling different numbers of variables to screen for the best combination of variables (see Figure 2(a)). In this study, the SVM-RFE hyperparameter selection of 10 variables produced the most accurate model (AUC = 0.673, Figure 2(b)). Then, the random forest model was constructed to evaluate its classification and prediction performance (AUC = 0.72, Figure 2(c)). Also, based on the factors of the random forest model, the importance of the variables were ranked in the model (see Figure 2(d)). Furthermore, univariate and multivariate logistic regression analyses were applied to identify factors that independently predicted the outcome (see Table 2). The results indicated that factors such as female, advanced age, sarcopenia, alcohol consumption, history of diabetes, anaemia, and depression were independent risk factors for cognitive impairment patients with gallstones (*P* < 0.05). The variables obtained from the screening were modelled in a multifactorial logistic regression prediction model based on a preset filter of *P* values.  Figure 2(e) displays that the model had AUCs of 0.779, 0.767, and 0.775 for the training group, the test group, and the whole cohort, respectively.  Figure 3(a) shows the relationship between the penalty coefficient log (lambda) and the variables retained by the model in the Lasso regression analysis. A total of 11 variables were filtered out based on the lambda.min value corresponding to the smallest loss value loss (see Figure 3(b)).  Figure 3(c) presents the names of these 11 variables and the corresponding coefficients. PCA for unsupervised cluster analysis was applied for these 11 variables. It was found that these 11 variables could be well differentiated for the presence or absence of cognitive impairment in patients with gallstones (see Figure 3(d)). The variables screened by lasso analysis were used to construct a multifactorial logistic prediction model to assess the predictive performance of the model in the validation set (AUC = 0.778, Figure 4(a)). This logistic regression model was constructed with the best predictive performance. Thus, this model was used for further follow-up analyses.

### 3.3. Clinical Visualisation Prediction Tool Construction

Based on logistic regression prediction models, a nomogram was plotted in R for the 11 characteristic variables obtained from the lasso analysis screening (see Figure 5). In this constructed model, gender, age, sarcopenia, history of alcohol consumption, diabetes, anaemia, and depression were found to be statistically significant difference factors associated with the development of cognitive impairment (*P* < 0.05, Table 3).

### 3.4. Nomogram Validation

The calibration curve assessing the predictive accuracy of the nomogram showed good agreement between the constructed model's prediction of cognitive impairment prevalence in patients with gallstones and the true observation (see Figure 4(b)). The ROC curve revealed that the constructed logistic regression model had AUCs of 0.787, 0.778, and 0.785 in the training group, the test group, and the whole cohort, respectively. In addition, the C-index of the model's predictions was also calculated for the three groups, at 0.787 (95% CI, 0.723-0.852), 0.778 (95% CI 0.778 (95% CI, 0.674-0.882), and 0.785 (95% CI, 0.73-0.839) (Table 4). These results indicate that the constructed nomogram had good predictive power. Moreover, the DCA revealed that the constructed model had a good level of clinical application and safety (see Figure 6). The results confirm that the nomogram and DCA can be tailored to patient needs and characteristics to help healthcare providers make better clinical decisions and provide a basis for safety and reliability for individualised interventions.

## 4. Discussion

In this study, four models were evaluated and compared to predict cognitive impairment in patients with gallstones. By comparing the predictive performance of each model or method, the best method was selected for model construction. Consequently, the clinical computational tool nomogram was drawn.

The results indicate that a multifactor logistic regression model based on 11 factors screened by LASSO regression analysis had the best predictive performance. These 11 factors were gender, age, education, place of birth, history of alcohol consumption, abdominal circumference, sarcopenia, diabetes, anaemia, depression, and PSQI. Based on the constructed logistic regression model, gender, age, history of alcohol consumption, sarcopenia, diabetes, anaemia, and depression were considered to be the factors associated with the development of cognitive impairment in patients with gallstones. The nomogram was built as a predictive tool for the development of cognitive impairment in patients with gallstones based on the best model constructed for the predictors. The accuracy of the model was further validated in both the training and test groups. The level of safety and reliability of the model was also evaluated in clinical applications. This predictive model was developed to assist healthcare providers in predicting the onset of cognitive impairment in patients with gallstones in advance based on risk factors. Thus, this model can help them provide appropriate and timely care, support, and treatment for patients.

This study suggests that female gender, advanced age, alcohol consumption, history of diabetes, sarcopenia, anaemia, and depression are all risk factors for developing cognitive impairment in patients with gallstones. The correlation between these factors and cognitive impairment has also been explored in several previous studies [10–12, 30]. The known risk factors for gallstone are female gender, increasing age, and metabolic syndromes such as obesity and overnutrition [1, 31–34]. Interestingly, Langa et al. showed that the risk of cognitive impairment increases with age and appears to be higher in men than in women [30]. Our findings also suggest that advanced age is a risk predictor for the development of cognitive impairment. However, our study found that female patients with gallstones were more likely to develop cognitive impairment than their male counterparts. This finding might be related to the fact that women are more likely to develop gallstones. Gallstones can lead to anorexia, whereby patients suffer from weight loss and malnutrition [3]. Malnutrition or mineral deficiencies are also found to be playing a role in the formation of gallstones [33, 35]. In addition, several previous studies have pointed out malnutrition as an independent risk factor for the development of sarcopenia [4, 5]. Consistent with our findings, sarcopenia is also reported to be a risk factor for cognitive impairment and cognitive impairment [6, 7]. Thus, cognitive impairment may exacerbate anorexia and further lead to malnutrition, perpetuating a vicious cycle of the disease. In summary, there seems to be a complex interaction between gallstones, malnutrition, sarcopenia, and cognitive impairment.

Frequent and heavy alcohol consumption is found to alter brain function, resulting in reduced cognition and even neurodegenerative diseases [36, 37]. Moreover, excessive alcohol consumption can also lead to mineral and vitamin deficiencies such as magnesium and folic acid deficiencies [38, 39]. Deficiencies in haematopoietic trace elements may cause anaemia. This is important since it has been shown that cognitive impairment is associated with anaemia [40]. This study also revealed that alcohol consumption was a significant predictor of developing cognitive impairment in patients with gallstones. Diabetes has also been found to be associated with cognitive impairment. Previous studies indicate that people with diabetes, especially those with poor blood sugar control, are at higher risk for developing cognitive impairment [41]. Another systematic review that included seven clinical studies came to similar conclusions, and they recommended testing and controlling patients' blood sugar to prevent or delay cognitive impairment [42].

It is also known that depression is an important cause of cognitive impairment [43]. Interestingly, loneliness was reported as an important factor in older patients for depression, contributing to the progression of cognitive impairment [44]. Social support is found to reduce depression in older people. Family support, in particular, is known to have a greater impact on depression in older people living in Asian communities [45]. Therefore, support groups such as family and friends can play an important role in improving elderly people's mental well-being by actively interacting and communicating with them [46]. Early detection and treatment are critical for optimal clinical outcome in patients with cognitive impairment, especially those at high risk of cognitive impairment. Potentially effective interventions for patients with cognitive impairment include meals with caregivers, family-style meals, soothing mealtime music, formal and informal caregiver support, and multifunctional interventions [47]. In summary, health workers can employ a myriad of preventive and therapeutic measures to alleviate the illness and enhance the psychological care of patients at risk of cognitive impairment. The current treatment of gallstones relies mainly on surgery [1]. Cognitive impairment often prevents patients from undergoing surgery [8]. Thus, it is crucial to screen for, prevent, and treat cognitive impairment in patients with gallstones as early as possible.

Cognitive impairment is known to be a significant challenge for society and families. In order to properly address this challenge, in this study, we developed and validated a nomogram to predict the risk of cognitive impairment in patients with gallstones. This is the first nomogram to be constructed for the prediction of cognitive impairment in patients with gallstones, thus offering the possibility of individualised screening. Furthermore, this model allows for the early intervention and treatment of patients, potentially reducing the risk of exacerbation of cognitive impairment. Analysing the net benefit to patients also revealed that the model has good levels of clinical application and safety. The clinical prediction model, based on the present statistical characteristics, has satisfactory classification performance and clinical application. However, there were some limitations in this study. Firstly, the prediction model lacked external data sets for validation. The research results show that the performance of logistic regression model is better than that of random forest. It may also be because the amount of data does not meet the requirements. Moreover, conducting a multicentre prospective study would allow us to obtain a higher level of evidence for clinical application and provide better generalisable findings. Secondly, the study should have been further developed to include more cognitive impairment-related characteristics, for example, by adding a multimodal database. Third, the evaluation result of C-index is low, so it is difficult to prove that it is an accurate prediction. Also, the model should be further optimised through further multicentre studies and increased sample size. In future work, investigating the ease with which the model can be mastered by health professionals and accepted by patients in clinical practice might prove important.

Both early intervention and social support play a vital role in reducing the risk of cognitive impairment in older patients, the consumption of valuable healthcare resources, and the cost to society. The constructed predictive model allows us to screen patients with gallstones and at high risk of cognitive impairment. Surgeons can employ the nomogram to make appropriate and timely decisions about the indications for surgery. Prediction results also enable healthcare professionals to intervene with families and the community for patients at high risk of cognitive impairment in the early stages. These efforts might also help to further increase patient compliance, assist healthcare professionals to better manage patients with gallstones, and ultimately improve their overall health status and quality of life.

## 5. Conclusion

In summary, this study developed and validated a highly accurate nomogram for predicting the risk of cognitive impairment in patients with gallstones. The constructed model provides a clinical basis for individualised diagnosis and treatment of patients with gallstones who are at risk of developing cognitive impairment. The nomogram was constructed to assist physicians in determining the need, suitability, and optimal time for surgery in patients with gallstones. It might also help caregivers and family members better monitor patients' conditions and ultimately improve the quality of life of patients with gallstones.

## Figures and Tables

**Figure 1:** Flow chart of this research programme.

**Figure 2:** Multiple model training prediction results are shown along with the selection process and prediction feature factor screening. (a) Line graph of the process of hyperparameter selection for the support vector machine model. The horizontal axis is the number of features incorporated into the support vector machine model, and the vertical axis is the accuracy of the corresponding model's classification predictions. The model has the highest prediction accuracy in the training group when 10 features are included, with an accuracy of 0.747. (b) Based on the relationship between the model performance and the corresponding hyperparameters, the 10 features corresponding to the best model performance are included in the support vector machine model for training, and its classification prediction performance is evaluated in the test group. AUC = 0.673; (c) the ROC curve shows that the random forest model has good classification performance in the test group (AUC = 0.72). (d) This bar graph shows the importance ranking of each factor incorporated in the random forest model modelling. Pittsburgh Sleep Quality Index (PSQI); Quality of Life Questionnaire Core 30 (QLQ-C30); (e) eight factors were obtained by single and multifactor logistic regression analysis. The ROC curve shows that the logistic regression prediction model constructed based on these eight factors had good classification prediction ability in both the training group (AUC = 0.779) and the test group (0.767).

**Figure 3:** The Lasso regression model is based on a default 10-fold crossvalidation for the process of variable screening and initial assessment. (a) This graph shows the relationship between the penalty coefficient log (lambda) and the retained variables. The number of intersecting curves is the number of variables retained at that log (lambda) value. (b) Using the 10-fold crossvalidation method, the relationship between binomial deviance and log (lambda) is plotted. (c) This bar graph displays the names of the 11 variables selected and their corresponding coefficient values. (d) Scatter plot exhibits the unsupervised clustering of the 11 variables using PCA, which allows a good differentiation between the presence and absence of cognitive impairment in patients with gallstones. The pink dots represent patients without cognitive impairment, and the blue dots represent patients with cognitive impairment.

**Figure 4:** Model predictive power validation and assessment. (a) The ROC curve shows that the logistic regression model constructed from the variables screened by lasso regression has optimal predictive power. The AUCs were 0.787, 0.778, and 0.785 in the training, test, and whole cohorts, respectively; (b) calibration curve displays the predictive ability of the model for cognitive impairment prevalence in patients with gallstones. The dashed line represents the predictive ability of the model to show a 100% match under optimal expectations. The solid line represents the predictive ability that the trained model would exhibit in a real situation. The closer the solid and dashed lines are to each other, the better the predictive ability of the chosen model (*B* = 1000).

**Figure 5:** A predictive model was constructed using 11 variables screened by lasso regression, and a nomogram was created to calculate and predict the likelihood of cognitive impairment in patients with gallstones.

**Figure 6:** Clinical usability and safety of the model. Application of clinical decision analysis curves to assess the range of clinical applicability and safety of the model in predicting the likelihood of cognitive impairment in patients with gallstones.

**Table 1:** Demographic and clinical characteristics of patients with or without cognitive impairment.

Variables	Normal (*n* = 184)	Dementia (*n* = 110)	*P* value
Age (year)	67.85 ± 6.25	71.83 ± 7.40	<0.001^∗∗^
Sex			
Female	110 (59.78)	82 (74.55)	0.010^∗^
Male	74 (40.22)	28 (25.45)	
Heart rate (bpm)	78.70 ± 10.22	77.74 ± 8.87	0.412
BMI (kg/m^2^)	24.39 ± 3.11	24.11 ± 3.39	0.471
Waist (cm)	86.09 ± 8.50	93.58 ± 86.20	0.243
Sarcopenia			
No	169 (91.85)	76 (69.09)	<0.001^∗∗^
Yes	15 (8.15)	34 (30.91)	
Marital status			
Married	173 (94.02)	103 (93.64)	0.894
Single	11 (5.98)	7 (6.36)	
Education level			
Illiteracy	50 (27.17)	35 (31.82)	<0.001^∗∗^
Primary education or below	77 (41.85)	63 (57.27)	
Secondary education or above	57 (30.98)	12 (10.91)	
Homeplace			
Rural areas	76 (41.30)	56 (50.91)	0.109
Urban areas	108 (58.70)	54 (49.09)	
Smoking			
No	168 (91.30)	105 (95.45)	0.181
Yes	16 (8.70)	5 (4.55)	
Drinking			
No	181 (98.37)	97 (88.18)	<0.001^∗∗^
Yes	3 (1.63)	13 (11.82)	
Hypertension			
No	95 (51.63)	44 (40.00)	0.053
Yes	89 (48.37)	66 (60.00)	
Diabetes			
No	161 (87.50)	83 (75.45)	0.008^∗∗^
Yes	23 (12.50)	27 (24.55)	
Anemia			
No	165 (89.67)	85 (77.27)	0.004^∗∗^
Yes	19 (10.33)	25 (22.73)	
Exercise			
Less than 3 times a week	70 (38.04)	50 (45.45)	0.042^∗^
More than 3 times a week	50 (27.17)	16 (14.55)	
No	64 (34.78)	44 (40.00)	
Medical insurance			
Commercial insurance payment	174 (94.57)	104 (94.55)	0.994
Self-paying	10 (5.43)	6 (5.45)	
Depression			
No	120 (65.22)	47 (42.73)	<0.001^∗∗^
Yes	64 (34.78)	63 (57.27)	
PSQI	6.47 ± 3.77	7.81 ± 3.39	0.003^∗∗^
Social Impact Scale	62.43 ± 8.54	62.22 ± 7.04	0.823
Total score QLQ-C30	56.69 ± 11.91	55.38 ± 10.87	0.347

^∗^ *P* < 0.05; ^∗∗^*P* < 0.01. Values are mean ± SD or number (percents%). Pittsburgh Sleep Quality Index (PSQI).

**Table 2:** Uni- and multilogistics regression analysis.

Variables	Uni-logistics regression			Multilogistics regression		
	*β*	Odds ratio (95% CI)	*P* value	*β*	Odds ratio (95% CI)	*P* value
Sex	-0.678	0.508 (0.298-0.847)	0.011	-0.831	0.436 (0.211-0.86)	0.020
Age	0.084	1.088 (1.05-1.129)	*P* ≤ 0.001	0.052	1.053 (1.008-1.102)	0.022
Heart rate	-0.010	0.99 (0.966-1.014)	0.411			
BMI	-0.027	0.973 (0.902-1.047)	0.470			
Waist	0.003	NA	0.408			
Sarcopenia	1.617	5.04 (2.636-10.049)	*P* ≤ 0.001	0.982	2.669 (1.244-5.838)	0.012
Marital status	0.067	1.069 (0.383-2.801)	0.894			
Education level/illiterate						
Primary education or below	0.156	1.169 (0.679-2.024)	0.575			
Second education or above	-1.201	0.301 (0.137-0.627)	0.002			
Homeplace	-0.388	0.679 (0.421-1.091)	0.110			
Smoking	-0.693	0.5 (0.16-1.319)	0.189			
Drinking	2.090	8.086 (2.533-35.887)	0.001	2.251	9.498 (2.153-54.008)	0.005
Hypertension	0.471	1.601 (0.995-2.594)	0.054	0.141	1.151 (0.648-2.041)	0.630
Diabetes	0.823	2.277 (1.232-4.245)	0.009	0.960	2.611 (1.305-5.296)	0.007
Anemia	0.938	2.554 (1.337-4.953)	0.005	0.989	2.69 (1.199-6.14)	0.017
Exercise/less than 3 times a week						
More than 3 times a week	-0.803	0.448 (0.224-0.862)	0.019	-0.691	0.501 (0.226-1.075)	0.081
No	-0.038	0.962 (0.567-1.633)	0.887	0.056	1.057 (0.574-1.949)	0.858
Medical insurance	0.004	1.004 (0.333-2.784)	0.994			
Depression	0.922	2.513 (1.553-4.099)	*P* ≤ 0.001	0.923	2.517 (1.293-4.997)	0.007
PSQI	0.102	1.107 (1.036-1.186)	0.003	0.017	1.017 (0.927-1.116)	0.714
Social Impact Scale	-0.003	0.997 (0.967-1.027)	0.822			
Total score QLQ-C30	-0.010	0.99 (0.969-1.011)	0.347			

*β* is the regression coefficient.

**Table 3:** Prediction factors for prevalence of cognitive impairment.

Variables	*β*	Odds ratio (95% CI)	*P* value
(Intercept)	-5.455	0.004 (0-0.127)	0.002
Sex	-0.777	0.46 (0.214-0.953)	0.041
Age	0.050	1.052 (1.005-1.102)	0.030
Waist	0.004	NA	0.435
Sarcopenia	1.117	3.055 (1.391-6.894)	0.006
Education level (illiterate)			
Primary education or below	0.532	1.702 (0.875-3.375)	0.121
Secondary education or above	-0.627	0.534 (0.174-1.557)	0.259
Homeplace (rural areas)	-0.173	0.841 (0.45-1.566)	0.585
Drinking	2.247	9.456 (2.284-50.568)	0.004
Diabetes	1.005	2.733 (1.341-5.665)	0.006
Anemia	0.907	2.477 (1.099-5.682)	0.030
Depression	0.780	2.181 (1.117-4.336)	0.024
PSQI	0.027	1.027 (0.933-1.13)	0.585

*β* is the regression coefficient.

**Table 4:** C-index of the nomogram prediction model.

Dataset	C-index of the prediction model	
	C-index	The C-index (95% CI)
Training set	0.787	0.723-0.852
Validation set	0.778	0.674-0.882
Entire cohort	0.785	0.73-0.839

## Data Availability

The datasets generated and analyzed during the present study are available from the corresponding author on reasonable request.

## Abbreviations

DCA: Decision curve analyses
HAMD-17: Hamilton Rating Scale for Depression (17-item version)
LASSO: The least absolute shrinkage and selection operator
PCA: Principal component analysis
PSQI: Pittsburgh Sleep Quality Index
MMSE: Mini-Mental State Examination
CRD: Clinical Dementia Rating
SIS: The Social Impact Scale
EORTC: The European Organisation for Research and Treatment of Cancer
QLQ-C30: Quality of Life Questionnaire Core 30
SVM-RFE: Support Vector Machine-Recursive Feature Elimination
ROC: The receiver operating characteristic curve
AUC: Area under the curve.
